The article "A 360-Degree View: An Autobiographical Case Report" was published in 2021. Journal: Cureus.

# A 360-Degree View: An Autobiographical Case Report

**DOI:** 10.7759/cureus.20337

**Published:** 2021-12-10

**Authors:** Wafa Sohail

**Affiliations:** 1 Internal Medicine, Dr. Ruth K.M. Pfau Civil Hospital, Karachi, PAK

**Keywords:** tb – tuberculosis, psychological impacts, public health care, health awareness, diagnostic delay, communicable disease control, autobiographical case report

## Abstract

The disease burden of tuberculosis (TB) has been declining in the developed world but the goal of eradicating TB seems like a daunting task in the developing regions. Patients with unrecognized TB or those receiving inappropriate treatment pose the greatest risk to the global burden of the disease. The aim of this article is to share the first-hand experience of a doctor, the author, contracting TB and the associated psychological impact. This change in role from a doctor to a patient came as an enlightening experience for the author and would give an insight into the psychological aspect when planning to find effective ways in the fight to eradicate TB.

## Introduction

The tertiary care hospitals in South Asia have been able to serve well if not extraordinarily. Considering the high population rate and limited resources available, the enthusiastic interns, nurses, and residents work diligently on the front line to save lives. Those who are taught how to treat tuberculosis (TB) are the ones at the highest risk of catching the communicable disease [1]. Studies have shown that the incidence of occupational TB is fairly high in health care workers compared to those working elsewhere [1]. These government-funded hospital settings have become a seeding ground for the spread of TB.

Working in a tertiary care setting can be a challenging task at times. Due to a lower level of awareness among the masses, the emergency rooms may show some upsetting scenes. Preventable diseases often show up in their worst forms. It is heartbreaking to see patients struggling for life, for conditions that could be managed well with timely advice. Talking about TB, in particular, many patients seek medical advice due to complications of the disease unaware of the fact that their disease has been progressing slowly. Such undiagnosed cases make up the most number of cases [2]. These patients not only pose a risk of spreading TB to the family members, but they also put health workers at risk.

In this case report, the author shares her experience of contracting*Mycobacterium tuberculosis*, how she got diagnosed, and the psychological impact of the illness. Various studies have been done describing the pathophysiology of TB, complications associated with untreated infection, and side effects of the medications; however, the psychological impact on the patient seems to be underreported along with its effect on the disease outcome and health-related quality of life after treatment.

The article "A 360-Degree View: An Autobiographical Case Report" was published in 2021. Journal: Cureus.

## Case presentation

I was sitting on the couch, sipping a cup of hot chocolate on my day off, when an unusual sensation in the back of my throat caught my attention. It did not feel like a usual postnasal drip. The consistency felt different. I went to the restroom to spit it out and what I saw came as a rude shock. I was staring at fresh blood. Before I could recollect myself, there was a bout of cough, which made me throw up more and more blood. Soon I was trembling. My heart started racing like a horse. The sympathetic system came into action and the catecholamines were all over the place. The cough did not seem to stop, making it difficult for me to step out of the restroom. My brother came to check on me and was surprised to see blood on the nasal orifices. The gush of blood was so powerful that it found its way to the nasal cavity. Worrying about how my mother would react to this disturbing situation, I tried to calm down by having some water, and soon we left for the hospital.

This was about April 2020, when the coronavirus disease 2019 (COVID-19) pandemic was in full swing. Hospitals were taking measures to accommodate the rising number of COVID-19 patients. All elective surgeries were postponed. Outpatient clinics were running for selected patients triaged from the emergency room. I was assessed in the triage and was asked to return for an appointment the next day. Feeling relieved about not having to stay in the hospital, I spent the rest of the day in my room. I began to think about all the possible causes of hemoptysis. I remember coming up with differentials in my mind just like we do on grand rounds but here I was thinking of all the benign causes because I was not prepared for the news yet. The next day we reached the hospital for the scheduled appointment. Having to walk a few steps to reach the doctor’s office, I started feeling short of breath. By this time I was sure that something serious was coming my way. It is rightly said that willpower is the driving force of the outcome of a patient’s illness. And as I was losing hope, I was losing my strength to bear all that was happening. The chest x-ray was done right away and was soon available for my pulmonologist to look at. He told me he could see a cavity in my lung. It was near the bronchus and was the most probable cause of hemoptysis. Considering my exposure as a doctor, TB was the most probable diagnosis and relevant tests were ordered. All of a sudden my symptoms from two months back started to make sense.

The article "A 360-Degree View: An Autobiographical Case Report" was published in 2021. Journal: Cureus.

I remember now that I had to consult a physician for flu-like symptoms that made me lose my appetite. I would feel weak and lethargic most of the time. The physician attributed my symptoms to viral asthenia as all my tests for viral infections such as malaria and dengue fever turned out to be negative. Viral asthenia refers to a feeling of tiredness or weakness that stays after a person has fought a viral infection. After that incident, I was never as energetic as before. Always feeling tired. I attributed my symptoms to burnout and fatigue, which is common amongst health care workers. I wish I had taken it more seriously. The hemoptysis came to me as a blessing in disguise. If I never had that bleeding episode, my diagnosis would have been delayed even further, increasing the chances of complications. The calm and soothing gentle voice of my pulmonologist brought me back to the present; he was reassuring me not to feel sad about having TB, a common infection in our region. At that moment I realized how empty such words may seem for a patient. TB is certainly a common illness in our region but nobody is prepared for it. Nobody would ever want to have it. Until now, it was me counseling patients diagnosed with TB and answering all their concerns; telling them that we understand how they must be feeling, making them feel comfortable to ask any questions they may have regarding the disease. But being on the other side of the table was painful. I asked myself, did I actually empathize with what my patients were feeling, or was it just a sympathetic response? My heart ached as I collected my sputum sample for the TB test called Acid- Fast Bacilli (AFB) culture. We would have to order these sputum cultures quite frequently considering the disease burden. This time collecting a sample for myself was heart-wrenching.

Things did not seem to go my way but I was able to control my emotions well. Or maybe I was not ready to feel anything yet. The next few days I tried to keep myself busy in isolation as I waited for the results. Social media did not seem to appeal anymore. The thought of not being able to work was haunting me. I could not imagine myself sitting idle. Although not feeling so myself, I tried to stay calm for my family. It was after a week from my first visit to the ER that I started to feel low. Not just physically but emotionally as well. The preliminary report of the AFB culture showed mycobacterial growth and I was to start my medication for the duration of the next six to nine months. The wave of thoughts that flowed through my mind is painful to recall. How patients eagerly wait for an answer from their doctor regarding a diagnosis. Their feelings and emotions upon hearing the difficult news. And how they try to accept and cope up with the emotional turmoil. I could feel all that.

The article "A 360-Degree View: An Autobiographical Case Report" was published in 2021. Journal: Cureus.

Isolation can be one of the most difficult things one may have to go through. But it was in isolation that I realized that it can be enlightening too, a steering moment in one’s life. It gives an opportunity to detach from the hustle and bustle in order to think clearly. This is where emotional support comes into play. I was lucky enough to have my family around. My friends and family have always found me optimistic and this was the time I wanted to make sure that I proved them right. The stigma associated with TB is the cause of many problems associated with the diagnosis and treatment. I was lucky enough to be surrounded by people who were well aware. The single thought that brought me out of that dark zone was: what if the cause of my hemoptysis had turned out to be a malignancy? Shouldn’t I be grateful to have something that is completely curable? What could have I done if there was something serious?

Slowly and gradually I came at peace with myself, my diagnosis, and adjusted my life around it. Out of the dark zone. But the sadness prevailed for quite some time. I remember auscultating myself from time to time to find any signs of improvement. I could feel what my patients would have to go through. I could recall the faces of some of the patients admitted for the treatment of complications due to advanced disease. One such girl who was just seventeen years old cannot be forgotten. She was admitted under our care for parapneumonic effusion due to TB and needed a chest tube. As an intern, I got a chance to assist my attending in placing the chest tube. The happiness on the face of that young patient and her family cannot be described in words. Chest tube limits one’s mobility and can be uncomfortable at times but the relief on the patient's face was really rewarding. Such patients coming from low socioeconomic status do not have high expectations because of the limited resources.

This girl and many other patients whom I could recall made me count my blessings. I had a room where I could isolate myself whereas these people living in small homes cannot do so, putting others in the family at risk. I was able to seek advice and could start the treatment right away without worrying about the stigma. This was made possible by the kind attitude of my colleagues and the moral support of family and friends. I had access to the Internet where I could find new recipes to cook for myself to nourish my body. This not only helped me discover my love for cooking but also help me regain my health faster whereas some of my patients could hardly afford bread. It is an established fact that good nutrition has a role in better outcomes of TB, still many cannot afford to have proper meals. What I did have in common with these patients were some medication side effects. I experienced severe joint pains. My feet would swell up whenever I sat on my desk for a few hours. My skin tone turned one tone darker. I had acneform lesions all over my face. It seemed like my skin could possibly never return to normal and it decreased my confidence to some extent. But I was glad that I did not have nausea and vomiting and was able to keep the medication down. After almost a year, no sign of any side effect is visible. My chest is clear and luckily the x-ray shows that my lungs are as good as before the illness. But the impact this phase had on my life shall remain forever. 

The article "A 360-Degree View: An Autobiographical Case Report" was published in 2021. Journal: Cureus.

We have considerable exposure to communicable diseases in South Asia as health care professionals but the risk has never undermined our passion to serve the community. In fact, after having it experience myself, the empathy towards patients has only grown stronger. I have become more grateful because the illness really made me count my blessings. Having to go through this experience in the early years of my profession will surely contribute to my passion for serving humanity.

## Discussion

Patients with unrecognized TB or those receiving inappropriate treatment pose the greatest to the global burden of TB. Historically considered a disease of the poor, TB has emerged as a global threat in the past few decades. The United Nations Sustainable Development Goals (SDGs) have set a target of ending TB by 2030 [3]. The available data shows that it would be a daunting task. The incidence of TB is falling at a rate of only 1.8% every year from 2016 [4]. It is, however, reassuring to see the incidence declining no matter how slow the progress may be. The reality is that the numbers fall short and TB is still the leading cause of death despite being a preventable and treatable cause. It is the second leading infectious killer after COVID-19 [5]. Figure 1 illustrates the annual Incidence of TB per 100,000 population by region. 

**Figure 1:** Annual worldwide tuberculosis incidence (per 100,000) by region, 2017 Figure Source: CDC; MacNeil A et al., 2019 [6]

Although considered a global health concern, TB cases are found to be clustered in low to middle-income regions struggling with overpopulation, malnutrition, and low literacy rates as shown in Figure 1. Southeast Asia and Africa account for two-thirds of the disease burden. Health-related quality of life after TB improves significantly with timely management of the disease, though the psychological impact of the disease has been seen to linger on for a while. According to Na Guo et al., this impact would worsen with delays in diagnosis and inappropriate treatment [7]. Delay in diagnosis not only increases the chances of complications but also increases the economic burden on the family. Low-income countries are, therefore, still fighting this crippling infectious disease due to the lack of awareness and social stigma associated with the disease. Oftentimes their economic status doesn’t allow them to seek care and may end up in the emergency room when the disease has already progressed. Those who do seek health advice in these under-served regions may often be misdiagnosed. Delay in diagnosis is another major factor associated with increased mortality. A study from South Asia reports an average delay of 55.3 days from the onset of symptoms to seeking medical advice for the first time [2]. It was also found that patients visited multiple providers before reaching a diagnosis [2]. Lack of qualified health workers in rural areas is a major barrier to access to health care [2].

The article "A 360-Degree View: An Autobiographical Case Report" was published in 2021. Journal: Cureus.

Compared to modern medicine, reliance on traditional medicine is another noteworthy factor in under-served countries [8]. Mistrust in the health care system is a notifiable barrier in adopting modern medicine and over-reliance on traditional medicine [8]. Patients consider traditional medicine as a safer option compared to advanced medical regimens. Medication side effects have been well reported [9]. it is important to spread awareness regarding the effectiveness of medication by emphasizing the fact that most of them are well tolerated and side effects are completely absent after completion of treatment [9]. *Mycobacterium tuberculosis *has the potential to affect any organ of the body and those who do not seek treatment for a long time may present with a systemic response to inflammation i.e. septic shock. Although pulmonary TB is the most common presentation, TB of other organs is also commonly seen in low to middle-income countries. Hematogenous spread of TB to abdominal organs, bones, vertebral column, and brain is seen. Therefore, encouraging the private providers to order regular screening tests for TB will help in early diagnosis, preventing the patients from complications [10].

Malnutrition and TB are often discussed together and there is strong evidence in the literature that links the two [11]. The higher incidence of TB in malnourished and low socioeconomic populations also points towards a relationship between the two. It is also noteworthy to mention that the at-risk population lives in overcrowded spaces with poor ventilation and sanitation. The World Health Organization’s agenda for this decade includes ending hunger and achieving food security by the year 2030 [5]. They have also outlined the research priorities in order to find a causal link between nutritional supplementation and the outcome of TB [12]. According to a study, undernutrition is associated with poorer outcomes of TB. Those with a higher BMI (>18.5) showed a lower mortality rate compared to those with lower BMI [13]. By addressing nutrition as an important determinant of pathogenesis and outcome of TB treatment, the health-related quality of life can be improved [14]. The genetic component linked with the pathogenesis of TB is less studied but has been well reported by a study [15]. According to a study, genetics has a role to play in the pathogenesis of TB, and studies at the genetics level may help in developing a successful vaccine [15].

The article "A 360-Degree View: An Autobiographical Case Report" was published in 2021. Journal: Cureus.

Although a completely curable illness, TB has a lingering impact on a patient’s life. TB-related disabilities, medication side effects, or the psycho-social impact have been studied. TB-related disabilities include respiratory impairment, mental health disorders, neurological impairment, and ophthalmic complications. These effects are mostly associated with multi-drug-resistant TB and are well reported. What seems to be underreported is the impact of TB on the mental health of patients. According to a study by Alene et al. [16], the prevalence of mental health impairment is found to be significantly high and they reported an incidence of 21.9% for mental disorders, second after respiratory impairment which was reported by 33.1% of patients. Depression, anxiety, post-traumatic stress disorder, and psychosis were seen among TB patients. The incidence was found to be higher in low to middle-income countries. Identifying the red flags at the beginning of treatment and timely referral of patients for a psychological evaluation would lead to better health-related quality of life [17].

The stigma associated with TB is an important determinant of the negative impact on a patient’s health. Delay in seeking treatment due to the fear of being labeled, the psychological stress associated with the diagnosis of communicable infection, and the health-related quality of life; all contribute negatively to a patient’s mental health. This chronic infection has a profound effect on physical health. Data shows that physical health improves more quickly compared to mental health [1]. Therefore, specific emphasis should be laid on addressing the patient’s mental well-being. It is very important to provide adequate knowledge about the disease with emphasis on the fact that it is completely curable with proper treatment. Identifying psycho-social stressors and facilitating the patient in coping with them can have a profound impact on the disease outcome.

The article "A 360-Degree View: An Autobiographical Case Report" was published in 2021. Journal: Cureus.

## Conclusions

Often times we are struck by the very thing we are scared to face. No matter how much we try to protect ourselves, if something is bound to happen, it will happen. This is what my diagnosis taught me. Working as a doctor in a region endemic to TB, I have always been well aware of the risk of contracting the disease. Having said that, it never undermined my passion to serve, nor did I let that become a hindrance in patient care. In fact, I have been actively involved in taking care of some of the very sick patients with TB. My motivation has only grown stronger after recovering from illness. Although, the diagnosis came to me as a blow, and going through the treatment was distressing, it has given me a clearer perspective regarding the true feelings of a patient fighting illness and the unpredictability of life in general. It has taught me to be less stringent about how I want things to be, leaving room for unprecedented situations. The diagnosis did shake me to the core but it proved to be an enlightening experience. It showed me the lows that patients may go through and taught me to stay hopeful that all will be well in the end. After all, hope must not die!

A commendable amount of work is being done for the fight against TB. Yet there is a lot more that needs to be done. This experience brought by a change in role from a doctor to a patient gave me a 360-degree view. It has increased my motivation to work on a community level. Our goal to eradicate TB cannot be achieved without running campaigns to spread awareness among people and my experience has only ignited the fire to do so. I feel like I am able to speak more passionately about it and I am using it to serve the cause. Let's keep striving to eradicate TB.
